This article has been retracted.

# Effects of Ultrasound Contrast Agent-Mediated Nerve Growth Factor on Apoptosis of Retinal Ganglion Cells in Mice with Glaucoma

**DOI:** 10.1155/2021/6084496

**Published:** 2021-11-27

**Authors:** Yan Ke, Lina Huang, Bingheng Chen, Jing Sima, Jiaguo Cao, Qiang Li

**Affiliations:** ^1^Aier Eye Hospital Group, Changsha, Hunan 410015, China; ^2^Shenzhen Aier Eye Hospital Affiliated to Jinan University, Shenzhen, Guangdong 518000, China; ^3^Department of Ophthalmology, Shenzhen People's Hospital, (The Second Clinical Medical College, Jinan University; The First Affiliated Hospital, Southern University of Science and Technology), Shenzhen, Guangdong 518020, China

## Abstract

With an increasing incidence in recent years, glaucoma (GL) has gradually become a global public health problem for humans of all ages. Nerve growth factor (NGF) eye drops, with well-documented stable effect in the treatment of GL, can be potentiated by the administration of NGF drugs via ultrasound contrast agent (UCA). This study analyzed the efficacy of NGF+UCA on GL mice and the influencing mechanism on retinal ganglion cells and further explored the pathological changes of GL mice under different UCA irradiation duration. In this study, we established GL mouse models and treated the mouse with NGF+UCA. The effect of NGF+UCA on intraocular pressure in mice was observed; the flash visual evoked potential of mice was compared; the changes of retinal structure, inflammation index, and oxidative stress index were observed, and autophagic protein levels were tested. Finally, the influence of UCA irradiation duration on GL symptoms was observed. The results showed that the intraocular pressure of mice decreased greatly, while their flash visual evoked potential and nervous layer of retina increased, and their ganglion cells showed stronger proliferation activity and weaker apoptosis and autophagy, indicating that UCA-mediated NGF can strongly improve the pathological condition of GL mice. In addition, PI3K/AKT pathway-associated proteins were inhibited in retina under the intervention of NGF+UCA, which further suggests that the influence of UCA-mediated NGF on GL is achieved by inhibiting autophagy of retinal ganglion cells and enhancing their apoptosis via the PI3K/AKT signaling pathway. Moreover, we found that in the treatment of GL, three weeks of UCA irradiation and six weeks caused no significant difference in the pathological manifestations and ganglion cells of mice, while after six weeks of irradiation, the level of NLRP3 in mice increased. In conclusion, UCA-mediated NGF can significantly improve the pathological condition of GL mice and improve the apoptosis of retinal ganglion cells by inhibiting autophagy, which is associated with the inhibition of the PI3K/AKT signal pathway. In terms of selection of UCA irradiation duration, three weeks of irradiation is enough to yield good clinical results.

## 1. Introduction

Glaucoma (GL), as an ophthalmic disease with fast onset and great harm in clinic, is very common among the middle-aged and elderly [1]. According to the survey, there are approximately 900,000 new cases with GL worldwide each year, with an emerging trend of the disease at younger ages [2]. The incidence of GL has increased by approximate 6-10 times since 2010, and researchers believe that it will become a global public health problem in all age groups as its incidence continues to rise [3]. GL is mainly induced by the imbalance of intraocular pressure (IOP), which has serious damage to various parts of the eyeball [4]. It is usually pathologically manifested as optic atrophy and vision loss, and over 70% of patients with GL have gone blind due to improper or untimely treatment [5]. It is estimated that by 2030, the number of GL-related blindness could exceed 20 million worldwide [6].

At the current stage, the clinical treatment of GL is mainly aimed at reducing IOP with drugs or surgery [7]. However, lowering IOP alone cannot completely hinder the development of GL. One study has pointed out that some patients with GL still had progressive nerve injury and obvious abnormal apoptosis of retinal ganglion cells after IOP lowering therapy [8], which not only seriously threatens the prognosis and health of such patients but also greatly increases the incidence of GL recurrence and other types of retinopathy [9]. Therefore, lowering the IOP of patients is just the foundation for GL treatment, and paying attention to the nerve injury of retina is the key to treating it.

Ganglion cells are a kind of cells unable to regenerate spontaneously. Traditional nerve-related drugs can only protect undamaged nerve cells and tissues to a certain extent but are unable to promote the regeneration of the damaged nerves [10]. Nerve growth factor (NGF) member of the neurotrophin family and its ability to promote neuronal growth, myelin synthesis, nerve cell development, and other nerve repair have been repeatedly verified in clinical practice. In ophthalmic diseases, NGF has been recognized clinically to treat retinopathy and keratopathy as an eye drop drug [11]. However, due to the existence of blood-eye barrier, the concentration of drugs in the retina and optic nerve is low, resulting in low efficacy of neuroprotective drugs and limited range of application [12]. Ultrasonic contrast agent (UCA) is a clinical means of enhancing ultrasound imaging by wrapping small bubbles with lipids, proteins, and other substances. In recent years, it has been found that UCA can also be used as a new scheme for targeted drug delivery [13]. According to one study [14], UCA can produce temporary and reversible pores to increase the permeability of cell membrane, thus enhancing the effect of drug delivery. Currently, it has been found to have remarkable effects in treating various tumor diseases.

As confirmed earlier, NGF can exert a stable effect in treating GL. The innovation and significance of this study are to determine whether UCA-mediated NGF is feasible for the treatment of GL and how long an intervention is appropriate. Therefore, by preparing GL animal models, we analyzed the effect of UCA-mediated NGF on retinal nerves of patients with GL and further explored the impact of different irradiation duration of UCA on GL, with the goal of providing novel therapeutic ideas for future clinical treatment of GL and laying a reliable foundation for subsequent research.

## 2. Materials and Methods

### 2.1. Data about Animals

With the experimental animal license number of SYXK (Su) 2021-0029, 80 C57BL/6 mice (8-12 weeks old, 20-30 g) purchased from Zhongchong Xinnuo Biopharmaceutical Co., Ltd. (Taizhou) were fed adaptively at (20 ± 2)°C with 3 mice in a cage under a 12-12-hour light-dark cycle, and they were given free access to food and water.

### 2.2. Establishment of GL Models

Totally 60 mice were randomly selected to establish GL models, of which 10 mice received no treatment as controls and 10 were used as substitutes. After anesthesia, the corneal limbal conjunctiva was cut off at the superior temporal, inferior temporal, and superior nasal quadrants to separate the extraocular muscles and fascia. Subsequently, the superior scleral vein was cauterized with sterile pins, and the conjunctival sac was rinsed with gentamicin (Beijing Biolab Technology Co., Ltd.) after the veins became congested and white. After modeling, erythromycin eye ointment (Beijing Twinluck Pharmaceutical Co., Ltd.) was applied3 times a day for 3 days. An increase of IOP ≥ 10 mmHg 7 days after modeling was considered successful.

In the process of modeling, 5 rats died, and we randomly selected 5 rats from the substitutes for replacement. The success rate of modeling was about 91.7%.

### 2.3. Intervention Treatment

#### 2.3.1. Effects of NGF+UCA on GL Mice

Totally 30 GL model mice were selected and randomized into 3 groups: the NGF+UCA group: after the conjunctival sac was washed with iodophor, a needle tubing was used to penetrate into the vitreous cavity at 1-3 mm behind the corneoscleral limbus to inject 10 *μ*L NGF solution (Sinobioway Biomedicine Co., Ltd.) and microbubble suspension solution, after which the eyes of the mouse were coated with levofloxacin hydrochloride eye drops (Changchun Dirui Pharmaceutical Co., Ltd.) and hydrogel. Then, the coupling agent was applied to the skin of the palpebra superior, and the ultrasonic gene transfection instrument (Sonitron GTS, Japan) was placed at the application position for pulsed ultrasonic irradiation for 60 seconds, with a sound intensity of 0.5 W/cm^2^. The irradiation was performed 3 days per time for one week; the NGF group: intravitreal injection of NGF was performed according to the above scheme, and levofloxacin hydrochloride eye drops were given after completion; and the model group: the mice received no treatment.

#### 2.3.2. Selection of Intervention Duration with NGF+UCA on GL Mice

The remaining 30 GL model mice were randomized into three groups: the one-week group (the mice were treated with NGF+UCA as described above and irradiated with UCA for one week), the three-week group (the mice were treated with NGF+UCA as described above and irradiated with UCA for three weeks), and the six-week group (the mice were treated with NGF+UCA as described above and irradiated with UCA for six weeks).

### 2.4. Sample Collection

On the 5th day after the above operation, the IOP of mice in each group was measured, and then all rats were anesthetized. The fellow eye of each mouse was covered, and an acupuncture needle electrode was inserted under the periosteum at the midpoint of the eyes, with the grounding electrode placed behind the right ear, and the resistance of <10 k*Ω*. Both eyes of mice were examined by full-field white flash stimulation, and the superposition value of 100 responses was recorded. In addition, the flash visual evoked potential (FVEP), including latency and amplitude of P100 wave, was recorded with the electrophysiological system. Then all mice were executed by cervical dislocation, and their whole eyeballs were obtained. The retina was quickly separated, and the retinal tissue homogenate, which was made quickly in the ice bath, was stored in the refrigerator at -80°C for use. After corneal incision, the iris and lens tissues were extracted, and the thickness of retinal ganglion cell layer (GCL), retinal nerve fiber layer (NFL), and retinal nerve fiber layer (NFL) was evaluated under an optical microscope.

### 2.5. Enzyme Linked Immunosorbent Assay (ELISA)

Arterial blood (4 mL) was sampled from each mouse and centrifuged to obtain serum to determine the serum levels of NLRP3, IL-6, IL-8, TNF-*α*, malondialdehyde (MDA), and superoxide dismutase (SOD) by ELISA, strictly following the kit instructions. The NLRP3 ELISA kit was purchased from Beijing Baochen Biotechnology Co., Ltd. (Beijing, China); IL-6, IL-8, TNF-*α* MDA, and SOD ELISA kits were purchased from Nanjing Jiancheng Bioengineering Institute (Nanjing, China). Absorbance was determined at 450 nm, and the concentrations of the indicators in the serum were calculated according to the standard curve.

### 2.6. Expression of Proteins in Retina

Total protein obtained from retinal tissues was determined to understand its purity via bicinchoninic acid (BCA), and then the protein was treated by electrophoresis, membrane transferred, and incubation with primary antibodies LC3-II (1 : 1000, Cell Signaling Technology), Beclin (1 : 1000, Cell Signaling Technology), PIK3 (1 : 1000, Cell Signaling Technology), and AKT (1 : 1000, Cell Signaling Technology). On the next day, the primary antibodies were removed by washing the membrane, and the membrane was subjected to 2 h of incubation with secondary antibodies, followed by the development. Finally, the obtained image was analyzed by the ImageJ analysis software.

### 2.7. Determination of Retinal Ganglion Cell Activity

After retinal separation, the retinal ganglion cells were enzymatically digested for 45 min at 37°C. Upon the completion of digestion, the cells were pipetted, and the cell suspension was collected into the 24-well plate. After 6-7 days of culture, the cells grew a large number of protrusions. Retinal ganglion cells in each group were collected and digested to a 5 × 10^5^ cells/mL solution and transferred to a 96-well plate, followed by 4 h of incubation with 10 *μ*L CCK-8 solution in each well. Then, the optical density (450 nm) of each well was detected by a microplate reader. Additionally, retinal ganglion cells were obtained and trypsinized, and the cell apoptosis was determined by flow cytometry.

### 2.8. Statistical Analyses

SPSS 23.0 (Chicago, USA) was used for statistical analyses of the collected data. All data were presented by mean ± SD ($\bar{x}\pm \text{s}$), independent-samples *t* test was used to assess the differences between two groups, and comparisons among multiple groups were performed with one-way ANOVA followed by LSD post hoc test. *P* < 0.05 indicates a significant difference.

## 3. Results and Discussion

### 3.1. Comparison of IOP

Before intervention (at 7 d after modeling), the IOP of the NGF+UCA group, NGF group, and model group had no significant difference (*P* > 0.05) and was higher than that of the control group (*P* < 0.05). After intervention, the IOP was not statistically different between the NGF+UCA group and the control group (*P* > 0.05), which was lower than that of the NGF group and model group, and the IOP was higher in the model group compared with the NGF group (*P* < 0.05). In addition, compared with that before intervention, the IOP of the control group did not change significantly after intervention (*P* > 0.05) but decreased in the NGF+UCA group and NGF group while increased in the model group (*P* < 0.05, Table 1).

### 3.2. Comparison of FVEP

Among the four groups, the latency of P100 wave was the lowest in the control group and the highest in the model group, and the NGF+UCA group showed a lower latency of P100 wave compared with the NGF group (*P* < 0.05). In addition, among the four groups, the amplitude of P100 wave was found to be the highest in the control group and the lowest in the model group, and that in the NGF+UCA group was higher than that in the NGF group (*P* < 0.05, Figure 1).

### 3.3. Comparison of Retinal Structure

The thickness of NFL and IPL was not significantly different between the NGF+UCA group and control group (*P* > 0.05), which was higher than that in the NGF group and the model group (*P* < 0.05). The model group showed thicker NFL and IPL than the NGF group (*P* < 0.05). In addition, in terms of GCL thickness, the highest GCL thickness was found in the control group, followed in descending order by the NGF+UCA group, NGF group, and model group (*P* < 0.05, Figure 2).

### 3.4. Comparison of Inflammatory Factor Expression

Among the four groups, the highest levels of NLRP3, IL-6, IL-8, and TNF-*α* were found in the model group, followed in descending order by the NGF group, NGF+UCA group, and control group. Compared with the model group, the levels in the NGF group were significantly decreased, while those in the NGF+UCA group were obviously lower than those in the NGF group (*P* < 0.05, Figure 3).

### 3.5. Comparison of Oxidative Stress Injury

Among the four groups, the highest SOD level was found in the control group, followed in descending order by the NGF+UCA group, NGF group, and model group (*P* < 0.05); however, the reverse was true in terms of the level of MDA among the four groups (*P* < 0.05, Figure 4).

### 3.6. Comparison of Retinal Ganglion Cell Activity

Among the four groups, the strongest proliferation activity of ganglion cells was found in the control group, followed in descending order by the NGF+UCA group, NGF group, and model group (*P* < 0.05). The apoptosis rate was the highest in the model group, followed in descending order by the NGF group, NGF+UCA group, and control group (*P* < 0.05, Figure 5).

### 3.7. Expression of Autophagy-Associated Proteins

The levels of autophagy-associated proteins (LC3-II and Beclin) were the highest in the model group, followed in descending order by the NGF group, NGF+UCA group, and control group (*P* < 0.05, Figure 6).

### 3.8. Expression of the PI3K/AKT Pathway

The highest levels of PI3K and AKT proteins were found in the control group, followed by the NGF+UCA group, NGF group, and model group from high to low (*P* < 0.05, Figure 7).

### 3.9. Rescue Experiment

Ganglion cells in the NGF+UCA group were obtained and intervened by IGF-1, a PI3K/AKT signaling pathway activator, and then assigned to an IGF-1+NGF+UCA group to detect cell activity. The results revealed no significant difference in proliferation and apoptosis between the IGF-1+NGF+UCA group and the model group (*P* > 0.05, Figure 8).

### 3.10. Effects of UCA intervention Duration on GL Mice

According to the comparison results, no notable difference was found in IOP among one-week group, three-week group, and six-week group (*P* > 0.05). According to the determination results of FVEP, the three-week group and six-week group were not significantly different in latency and amplitude of P100 wave (*P* > 0.05). However, the lower latency of P100 wave in these two groups was lower, and the amplitude of P100 wave was higher compared with the one-week group (*P* < 0.05). In addition, the determination results of retinal structure showed that the NFL thickness differed insignificantly between the three-week group and the six-week group (*P* > 0.05), which was lower than that of the one-week group (*P* < 0.05). The highest GCL and IPL levels were found in the six-week group, followed in descending order by the three-week group and the one-week group (*P* < 0.05, Figure 9).

### 3.11. Effects of UCA Intervention Duration on Inflammation and Oxidative Stress Response of GL Mice

The determination results of inflammatory factors revealed similar IL-6, IL-8, and TNF-*α* levels in the three-week group and the six-week group (*P* > 0.05), which were lower than those in the one-week group (*P* < 0.05). The level of NLRP3 was not statistically different between the six-week group and the one-week group (*P* > 0.05), which was higher than that in the three-week group (*P* < 0.05). In addition, the determination results of oxidative stress injury showed that the three-week group and six-week group had no difference in SOD and MDA levels (*P* > 0.05), but compared with the one-week group, the SOD level in these two groups was higher while the level of MDA level was lower (*P* < 0.05, Figure 10).

### 3.12. Effects of UCA Intervention Duration on Ganglion Cells of GL Mice

No notable difference was found between the three-week group and six-week group in ganglion cell proliferation and apoptosis (*P* > 0.05), but compared with the one-week group, the proliferation activity of ganglion cells in these two groups was stronger, and cell apoptosis was weaker (*P* < 0.05). In addition, according to the autophagy-associated protein detection results, the three groups were not significantly different in LC3-II and Beclin levels (*P* > 0.05, Figure 11).

### 3.13. Discussion

In parallel with the population aging, ophthalmic diseases also show an increasing incidence in recent years [15]. GL, as a common and severe condition in the ophthalmology department, has no obvious characteristics in the early stage. The pathological features of this disease are severe damage to the eyeballs and surrounding tissues through the continuous increase of IOP, and the susceptibility to irreversible and serious damage to the visual nervous system [16]. NGF is a novel treatment scheme for various ophthalmic diseases, but its application effect still needs improvement [17]. It is shown that UCA can significantly improve the bioavailability and targeting ability of drugs [18]. Therefore, this study probed into the efficacy of UCA-medicated NGF on GL, which is of great significance for future clinical treatment of GL.

First, we compared the IOP among the four groups and found notably decreased IOP in mice in the NGF+UCA group and NGF group, indicating that both NGF+UCA and NGF can alleviate GL. Compared with the NGF group, the NGF+UCA group showed greatly improved IOP and better thickness of GCL, NFL, and IPL, suggesting the higher efficacy of UCA-medicated NGF in treating GL. One earlier study has confirmed that GL can cause serious damage to the intraocular retina due to the continuous increase of IOP, and the mechanism of such damage is strongly associated with accelerated apoptosis of ganglion cells [19]. NGF has been confirmed as a nutrient to promote the growth of nerve cells [20]. Treatment with it through eye drops can also alleviate GL to a certain extent. As the most common way of administration for ophthalmic diseases, eye drops can inhibit disease procession by dripping the drug into the conjunctival sac to be absorbed by the cornea, conjunctiva, and capillaries to enter the systemic circulation [21, 22]. However, during eye drop administration, the drug may be discharged from the body through the lacrimal passage and nasal cavity, so that the absorption of the drug is reduced, resulting in reduced efficacy that is not as significant as expected [23]. In addition, the dose of drugs delivered by eye drops is limited, while increasing the dropped dose cannot increase the bioavailability of the drugs but will enhance the drug toxicity instead [24]. In contrast, intravitreal injection is an effective way that can increase drug availability and improve the drug efficacy. In earlier studies, intravitreal injection for drug delivery has greatly improved the application effect of antivascular endothelial growth factor and glucocorticoid. Therefore, this study chose the glass intracavity injection for treatment. The results also showed that the effect in the NGF+UCA group was better. We speculate that this is due to the use of UCA, which exerts a more significant effect. With UCA, NGF can be injected into vitreous cavity in the form of microbubbles, which are subsequently blasted by ultrasound. As such, cell membrane permeability is increased, allowing NGF to be better absorbed by retinal tissues. On the other hand, it can activate the resistance of ganglion cells and reduce complications and adverse events, thereby improving the safety of treatment [25]. This can be confirmed by our detection results of FVEP, inflammatory factors, and oxidative stress injury. The detection results showed that the retinal damage of mice in the NGF+UCA group was greatly reduced. At present, UCA-mediated gene therapy has received unanimous clinical recognition with the advantages of strong specific targeting, high safety, and low immunogenicity. It can not only effectively mediate the molecular substances contained in it to achieve the target site but also further increase its ability to bind to cells, which has become a new direction for the treatment of many tumor diseases [26]. We speculate that in GL, due to the continuous increase in IOP, the physiological functions of normal cells in the optic nerve axon are affected, causing the accumulation of intracellular material and the swelling and degeneration of the axon. Meanwhile, the structure of the nerve axon is very disordered and the myelin sheath is dissolved and loosened to varying degrees [27]. Therefore, during intravitreal injection, the NGF molecules may be lost in large amounts due to structural changes or be absorbed and dissolved by other tissue components, preventing successful repair and regeneration of ganglion cells. While the encapsulation and protection of NGF by UCA can avoid the premature consumption of NGF and enhance cell membrane permeability to ensure that NGF has a better targeting effect and key parts, thereby enhancing the therapeutic efficacy.

It is well known that the pathological process of GL is strongly correlated with the damage of ganglion cells. To further understand the mechanism of NGF+UCA on GL, we detected the status of retinal ganglion cells in the four groups. The NGF+UCA group showed stronger proliferation of ganglion cells and weaker apoptosis, indicating that UCA-mediated NGF can promote the repair of ganglion cells and inhibit their apoptosis. According to autophagy-associated protein determination results, the NGF+UCA group showed weaker autophagy ability. Autophagy, as one of the main ways to accelerate the apoptosis of ganglion cells, is usually significantly enhanced after nerve injury [28]. Therefore, inhibition of autophagy is also a potential molecular pathway for the treatment of GL, which needs to be confirmed by subsequent studies. Moreover, we found through previous studies that PI3K/AKT is a signal pathway closely related to cell autophagy, and it is in an obvious activation state in cases with GL [29, 30]. Therefore, we also quantified PI3K/AKT protein in each group of mice. The results revealed decreased PI3K/AKT protein expression under the intervention of NGF+UCA, indicating that the signal transduction was inhibited, which may be one of the ways that NGF+UCA affected the autophagy of ganglion cells. Finally, through the rescue experiment, we found that after activating the PI3K/AKT signaling pathway in mouse ganglion cells intervened by NGF+UCA, the cell viability in these mice was completely consistent with that in the model group. The result indicates that activation of the PI3K/AKT signal pathway can reverse the influence of NGF+UCA, which confirms our view.

The above experiment results indicate the remarkable therapeutic effect of NGF+UCA on GL. In previous studies, Li et al. [31] carried out irradiation with UCA to mice with atherosclerosis for 2 weeks [32], and Huang et al. [33] treated mice with colon cancer with a total of six weeks of irradiation with UCA. At the current stage, the optimal UCA intervention duration for GL remains to be defined due to the absence of reliable research guidance. In order to further explore the influence of UCA irradiation duration on GL, we divided GL mice into three groups treated with different UCA irradiation duration and observed the differences among these groups. First of all, we found that UCA irradiation duration exerted no notable effect on IOP in GL mice. In terms of FVEP and retinal structure, there was no obvious difference between the three-week group and the six-week group, but both the two items of the two groups were better than those of the one-week group. Therefore, we preliminarily inferred that UCA could basically alleviate GL when its irradiation duration reached three weeks, while prolonging the irradiation had no significant effect on GL mice. Subsequently, the inflammatory reaction and oxidative stress reaction in mice were found to differ insignificantly between the three-week group and the six-week group, which were better than those of the one-week group. However, the level of NLRP3 in the six-week group was higher than that in the three-week group, which suggested that six weeks of irradiation with UCA may intensify the inflammatory reaction in mice instead. The reason behind it may be that UCA can temporarily open the cell membrane and increase cell permeability [34]. In the short term, it can increase the absorption of drugs by cells, but long irradiation may destroy the original stable structure of cells and deprive the protective ability of cell membrane, causing the initial sign of intensified inflammatory reaction. Of course, the specific reasons have yet to be confirmed by further experiments. Finally, the results of biological behavior test were basically consistent with the above: The three-week group and six-week group were not significantly different in ganglion cell proliferation and apoptosis, which further verified our view, whereas there was no difference in autophagy-associated protein expression among the three groups, which may be explained by the fact that the obvious inhibition on cell autophagy gives rise to no obvious visual difference in detection results.

The present study has preliminarily investigated the influence of UCA on GL, but there are still many limitations. For instance, the specific action pathway of NGF+UCA, its application effect in the human body, and the influence of different NGF dosages on efficacy are all still unclear, which will be the focuses and directions of our follow-up research.

## 4. Conclusion

UCA-mediated NGF can effectively improve the pathological condition of GL mice and enhance the apoptosis of retinal ganglion cells by inhibiting autophagy, the mechanism of which is associated with the inhibition of PI3K/AKT signal pathway. In terms of selection of UCA irradiation duration, three weeks of it is enough to deliver good results.

## Figures and Tables

**Figure 1:** FVEP. (a) P100 wave latency. (b) P100 wave amplitude. vs. the NGF+UCA group, ^∗^*P* < 0.05; vs. the NGF group, ^#^*P* < 0.05; vs. the model group, ^&^*P* < 0.05.

**Figure 2:** Retina structure. (a) GCL thickness. (b) NFL thickness. (c) IPL thickness. vs. the NGF+UCA group, ^∗^*P* < 0.05; vs. the NGF group, ^#^*P* < 0.05; vs. the model group, ^&^*P* < 0.05.

**Figure 3:** Inflammatory factors. (a) NLRP3 level. (b) IL-6 level. (c) IL-8 level. (d) TNF-*α* level. vs. the NGF+UCA group, ^∗^*P* < 0.05; vs. the NGF group, ^#^*P* < 0.05; vs. the model group, ^&^*P* < 0.05.

**Figure 4:** Oxidative stress injury. (a) SOD level. (b) MDA level. vs. the NGF+UCA group, ^∗^*P* < 0.05; vs. the NGF group, ^#^*P* < 0.05; vs. the model group, ^&^*P* < 0.05.

**Figure 5:** Comparison of retinal ganglion cell activity. (a) Proliferation of ganglion cells. (b) Flow cytometry. (c) Apoptosis of ganglion cells. vs. the NGF+UCA group, ^∗^*P* < 0.05; vs. the NGF group, ^#^*P* < 0.05; vs. the model group, ^&^*P* < 0.05.

**Figure 6:** Expression of autophagy-associated proteins. (a) Western blot map. (b) Level of LC3-II protein. (c) Western blot map. (d) Level of Beclin protein. vs. the NGF+UCA group, ^∗^*P* < 0.05; vs. the NGF group, ^#^*P* < 0.05; vs. the model group, ^&^*P* < 0.05.

**Figure 7:** Expression of the PI3K/AKT pathway. (a) Western blot map. (b) Level of PI3K protein. (c) Western blot map. (d) Level of Akt protein. vs. the NGF+UCA group, ^∗^*P* < 0.05; vs. the NGF group, ^#^*P* < 0.05; vs. the model group, ^&^*P* < 0.05.

**Figure 8:** Rescue experiment. (a) Proliferation of ganglion cells. (b) Flow cytometry. (c) Apoptosis of ganglion cells.

**Figure 9:** Effects of UCA intervention duration on GL. (a) Comparison of IOP. (b) P100 wave latency. (c) P100 wave amplitude. (d) GCL thickness. (e) NFL thickness. (f) IPL thickness. vs. the 1-week group, ^∗^*P* < 0.05; vs. the 3-week group, ^#^*P* < 0.05.

**Figure 10:** Effects of UCA intervention duration on inflammation and oxidative stress response of GL mice. (a) Comparison of NLRP3. (b) Comparison of IL-6. (c) Comparison of IL-8. (d) Comparison of TNF-*α*. (e) Comparison of SOD. (f) Comparison of MDA. vs. the 1-week group, ^∗^*P* < 0.05; vs. the 3-week group, ^#^*P* < 0.05.

**Figure 11:** Effects of intervention duration with on ganglion cells of GL mice. (a) Comparison of proliferation. (b) Flow cytometry. (c) Comparison of apoptosis rate. (d) Western blot map. (e) Comparison of LC3-II protein expression. (f) Western blot map. (g) Comparison of Beclin protein expression. vs. the 1-week group, ^∗^*P* < 0.05; vs. the 3-week group, ^#^*P* < 0.05.

**Table 1:** Comparison of intraocular pressure (mmHg).

	Before intervention	After intervention	*t*	*P*
NGF+UCA	32.47 ± 5.62	9.04 ± 2.22	12.260	<0.001
NGF	31.13 ± 4.97	23.63 ± 5.12^∗^	3.324	0.004
Model group	31.20 ± 8.36	38.63 ± 6.31^∗^^#^	2.243	0.038
Control group	8.88 ± 1.01^#&^	8.74 ± 0.78^#&^	0.347	0.733

Note: vs. the NGF+UCA group, ^∗^*P* < 0.05; vs. the NGF group, ^#^*P* < 0.05; vs. the model group, ^&^*P* < 0.05.

## Data Availability

The labeled dataset used to support the findings of this study is available from the corresponding author upon request.
